# Edge Constraint and Location Mapping for Liver Tumor Segmentation from Nonenhanced Images

**DOI:** 10.1155/2022/1248311

**Published:** 2022-03-09

**Authors:** Jina Zhang, Shichao Luo, Yan Qiang, Yuling Tian, Xiaojiao Xiao, Keqin Li, Xingxu Li

**Affiliations:** ^1^College of Information and Computer, Taiyuan University of Technology, Taiyuan, China; ^2^Department of Computer Science, State University of New York, New Paltz, New York 12561, USA

## Abstract

As there is no contrast enhancement, the liver tumor area in nonenhanced MRI exists with blurred edges and low contrast, which greatly affects the speed and accuracy of liver tumor diagnosis. As a result, precise segmentation of liver tumor from nonenhanced MRI has become an urgent and challenging task. In this paper, we propose an edge constraint and localization mapping segmentation model (ECLMS) to accurately segment liver tumor from nonenhanced MRI. It consists of two parts: localization network and dual-branch segmentation network. We build the localization network, which generates prior coarse masks to provide position mapping for the segmentation network. This part enhances the ability of the model to localize liver tumor in nonenhanced images. We design a dual-branch segmentation network, where the main decoding branch focuses on the feature representation in the core region of the tumor and the edge decoding branch concentrates on capturing the edge information of the tumor. To improve the ability of the model for capturing detailed features, sSE blocks and dense upward connections are introduced into it. We design the bottleneck multiscale module to construct multiscale feature representations using kernels of different sizes while integrating the location mapping of tumor. The ECLMS model is evaluated on a private nonenhanced MRI dataset that comprises 215 different subjects. The model achieves the best Dice coefficient, precision, and accuracy of 90.23%, 92.25%, and 92.39%, correspondingly. The effectiveness of our model is demonstrated by experiment results, and our model reaches superior results in the segmentation task of nonenhanced liver tumor compared to existing segmentation methods.

## 1. Introduction

According to the latest global cancer data released by the International Agency for Research on Cancer (IARC) of the World Health Organization, the number of deaths from liver cancer in 2020 ranks fourth in the world [1]. The diagnosis and treatment of liver cancer have always been the priority and difficulty of medical research. Liver tumor is a significant biomarker for the diagnosis of liver cancer, and accurate segmentation of liver tumor can greatly increase the detection rate of liver cancer [2]. However, the current segmentation of liver tumor is manually segmented by radiologists on a large number of MRI images slice by slice. The results of segmentation depend on the clinical knowledge and experience of the radiologist which is highly subjective and time-consuming [3]. Using deep learning technology to automatically segment liver tumor can avoid misdiagnosis caused by the subjective differences of physicians, speed up the screening of liver tumor, and lay the foundation for clinicians to accurately diagnose and formulate reasonable treatment plans. The model which automatically segments liver tumor can play a crucial role in the diagnosis and treatment of liver cancer.

In the clinical diagnosis of liver tumor, gadolinium-based contrast agents are usually injected into patients to enhance the contrast between the tumor and the surrounding organs [4]. Unfortunately, gadolinium-based contrast agents also bring many dangers: (1) the elements contained in the contrast agent may have specific toxic effects on the liver and kidney functions of the human body [5]; (2) standard clinical protocols usually require multiple MRI collections before and after contrast injection; this intermittent multiple collection takes more than twice the time of CT collection [6]; and (3) the use of contrast agents demands more medical resources (the extra equipment and labor) [7]. Segmentation of liver tumor in nonenhanced MRI images (without contrast agents) can eliminate the risk of injection of contrast agents; at the same time, it also reduces the detection time of patients and medical resource consumption. It has become an urgent clinical need to develop a kind of segmentation method without contrast agent [8]. Because of missing contrast enhancement, nonenhanced MRI images show extremely unclear tumor margins, the contrast with the surrounding tissues is low, and also, the anatomical structure is complicated. Liver tumors are diverse in shape and size. The diameter of a small liver tumor is usually less than or equal to 2 cm, the diameter of a massive liver tumor can reach more than 10 cm, and automatic segmentation of a small tumor is still a challenging task [9]. The comparison of enhanced and nonenhanced MRI is shown in Figure 1. The pixel distribution of normal tissue and tumor in the data has a high degree of similarity, and it is extremely hard to precisely locate and segment tumor.

Most of the current liver tumor segmentation work is based on enhanced images. Liu et al. [10] proposed a residual attention U-Net (ResAttU-Net) to segment liver lesions in enhanced images. The model incorporated the residual blocks and skip-connection attention modules to dig deeper into the features associated with the lesion. This model achieved a Dice score of 89.52% for liver tumor segmentation. Chlebus et al. [11] developed a fully automatic method for liver tumor segmentation in CT images based on a 2D fully convolutional neural network with an object-based postprocessing step. This method was ranked third in the MICCAI 2017 second round of liver tumor segmentation challenge. Hong et al. [12] presented an automatic segmentation framework based on 3D U-Net, which incorporates dense connection and global detail optimization. The method first obtained the probability map of the liver from incorporating the dense connection U-Net. Then, the probability map was refined as an initial surface and a priori shape. A multiscale approach was employed by Kushnure and Talbar [13] to scale the perceptual field of convolutional neural networks (CNNs). The multiscale block was able to pull in global and local features at a much finer granularity level. This method obtained 84.15% Dice score in liver tumor segmentation task. Mo et al. [14] proposed a segmentation method based on graph learning. It was motivated by extracting modality-specific features and constructing the regional correspondence effectively between T1WI and T2WI. The above works are based on enhanced MRI or CT data. The tumor in the nonenhanced data is less distinguishable compared to the enhanced images, and it will inevitably result in poor segmentation results that directly transfer from these methods to the nonenhanced image data.

Although many researchers have proposed a series of effective segmentation methods, few of them are directly applied to nonenhanced images. Klimont et al. [15] designed a semiautomatic segmentation method for cerebral angiography based on deep learning. This method performed spatial alignment, denoising, and manual correction on brain CT with and without contrast to generate a binary mask. Then, they trained their model designed basing on the U-Net structure to perform blood vessel segmentation from noncontrast CT images. This semiautomatic segmentation method has two weaknesses. On the one hand, the data input to the model must undergo a series of tedious preprocessing steps. On the other hand, the quality of the labels in the data is poor. Xu et al. [16] used spatial correlation which represents different time and step sizes in cardiac images and the complementarity between quantization and segmentation as reference information. The integrated spatiotemporal features of myocardial infarction were extracted from 2D temporal sequence images (2D+T), and automatic segmentation of myocardial infarction without contrast agents was realized. This method is only suitable for dynamic image segmentation, such as dynamic heart image, but not for static image without spatiotemporal characteristics. In the field of liver tumor segmentation, Xiao et al. [17] proposed a radiological-guided GAN (radiomics-guided GAN). The radiomic characteristics of contrast-enhanced images were introduced into the discriminator as prior knowledge to guide the adversarial learning of the segmentation network to segment liver tumor from nonenhanced MRI images. This work is the first method to accomplish liver tumor segmentation on nonenhanced images, but the huge number of parameters makes generalization difficult in medical images with small amounts of data. Zhang et al. [18] introduced a kind of the relative entropy bias and proposed two tumor detection strategies to identify the tumor location. They used the tumor features visible in the enhanced image as a guidance information to assist the segmentation task in the nonenhanced image. It was a weakly supervised segmentation method; the Dice and recall of this method are 83.11% and 85.12%, correspondingly. Both of the above methods promote segmentation by introducing different tumor-related features as guides. Zhao et al. [19] proposed a united adversarial learning framework for simultaneous liver tumor segmentation and detection using multimodality noncontrast MRI. However, existing works have ignored the value of tumor edge information in enhancing segmentation accuracy; at the same time, the difficult of tiny tumor segmentation has not been well addressed.

Different from these existing methods, we build a liver tumor segmentation model on the basis of edge constraints and location mapping, named edge constraint and localization mapping segmentation model (ECLMS). It consists of localization network and dual-branch segmentation network, which is used to segment liver tumors from MRI images without contrast agents. Inspired by Oda et al. [20], we design a dual-branch segmentation network. With task-independent decoders forming edge branch and main branch, these two branches efficiently exploit tumor features and edge features, individually, while enabling edge branch and main branch to promote each other for finer segmentation of tumor details. The SE block proposed by Hu et al. [21] learns channel-specific descriptors by global averaging pooling to exclude spatial dependencies. This descriptor is employed to recalibrate the feature map to highlight useful channels. This approach mines information along the channel direction, which is effective for classification, while for fine-grained image segmentation, the spatial information of pixels is more critical. Inspired by SE blocks, another spatial SE block (sSE) [22] is presented, which is “squeezed” along channels and “excited” spatially, and is more suitable for segmentation networks. We embed sSE block into the network, prompting the network to pay more attention to informative features and suppress unimportant ones. The diverse tumor morphology creates a challenge for intensive pixel-level prediction. Using multiscale of receptive fields to capture targets with large variations in shape is essential to improve the accuracy of tumor segmentation. In traditional convolutional networks, fixed-size convolutional kernels are usually used. It is difficult to represent each pixel with a single-scale feature. But multiperceptual fields of different sizes can expand the perceptual dimension of the network. To improve the segmentation accuracy of different-size tumors, especially small tumors, the bottleneck multiscale module (BMM) is introduced by us to capture features at different scales. Because background tissue with similar grayscale values as the tumor is deceptive and distracting to the model, segmentation networks on their own are still insufficient to accurately identify the tumor. A typical method to solve this problem is to utilize the classification network to identify the notable area in the image [23, 24]. However, the location maps generated directly by the classification network may only contain the discriminative regions related to the category, which is not enough to guide the generation of accurate segmentation masks. Some studies have proved that segmentation networks can effectively promote the performance of classification networks [25, 26]. Therefore, an additional localization network is brought to generate the location mapping of the tumor, which includes a segmentation network and a classification network. A segmentation network is first used to generate a coarse segmentation mask. Then, a classification network is applied to determine the correctness of the coarse segmentation mask and generate a location mapping. Finally, the location mapping is merged with the high-dimensional features in the middle of dual-branch segmentation network to alleviate the bias caused by inaccurate features so as to increase the learning ability of the segmentation network for low-contrast lesion regions. In summary, the contributions of this paper are as follows:

- We propose a novel edge constraint and location mapping for liver tumor segmentation model, so called ECLMS. This model can segment liver tumor from nonenhanced MRI. The final segmentation result (Dice) reaches 90.23%, which has superior performance
- Considering the complementarity between tumor and edge, we innovatively design a dual-branch segmentation network. And the sSE block is embedded in it to enhance the network's capability to capture the critical features. At the same time, the features of different layers and sizes in the encoder-decoder are fused by dense upward connections to enrich the shallow network features and alleviate the information degradation in the coding process. To the best of our knowledge, this is the first time that edge information is utilized in nonenhanced image segmentation to improve the segmentation accuracy of tumor
- We propose a bottleneck multiscale module (BMM) to extract features at different scales, while integrating the location mappings generated by the localization network to adapt the network for targets with diverse morphological sizes
- We construct a localization network for generating location mappings to alleviate the negative impact of inaccurate localization on segmentation results. It allows the network to concentrate more effectively on the tumor region and improves the segmentation performance

## 2. Related Work

### 2.1. Medical Image Segmentation

Biomedical data is increasing in volume thanks to advances in image acquisition methods. The automated analysis of these large-scale datasets presents new challenges for data-driven and model-based computational approaches. During the past few decades, medical image segmentation methods have mainly focused on developing algorithms, such as watershed [27], level set [28], statistical shape model [29], region growing [30], active contour model [31], graph cuts [32], threshold processing [33], and traditional machine learning methods [34], but these methods require manual extraction of tumor features. In the latest years, Deep Neural Networks (DNNs) have been widely implemented to learn increasingly complex feature hierarchies from processed data, thereby enabling multilevel abstraction. Specifically, DNNs exploit the property that many natural signals are compositional hierarchies (i.e., higher-level features are obtained by composing lower-level ones) [35]. Deep learning methods have made great breakthroughs in medical image segmentation. In the 2017 liver tumor segmentation challenge (LiTS), the automatic segmentation methods that submitted high scores almost all used the fully convolutional network architecture (FCNs), and its fully connected layers were replaced by convolutional layers [36]. The popular U-Net [37] was a variant of FCN, which consists of an encoder, a decoder, and a skip connection between them. Medical images have fuzzy boundaries and complex gradients, which need more high-resolution information. Because the internal structure of medical images is relatively fixed, the distribution of segmentation targets in the images is very regular and the semantics are simple and clear. Low-resolution features can provide structural information to identify targets. U-Net cleverly combines low-resolution information with high-resolution information. However, the parameters of its network are much smaller than those of most natural image semantic segmentation networks. As a result, U-Net can better adapt to medical images with scarce samples. Due to the good effect of U-Net in medical image segmentation, it has been widely used in various segmentation networks. Some common improvement methods include redesigning skip connection and adding dilated convolutions or residual connections. Schlemper et al. [38] introduced a soft attention-gated mechanism, an early application of soft attention ideas to medical image analysis. This mechanism is able to suppress the task-irrelevant part of network learning while enhancing the task-relevant features. The U-Net++ network proposed by Zhou et al. [39] set up U-Net sets of different depths and redesigned the skip connections. The redesigned skip connection allowed to acquire features at different levels and integrate them. This approach overcomes the unnecessary limitations in fusing features at the same scale but also increases the number of parameters exponentially. Inspired by this idea, we connect the deep features of the encoder to the shallow layer of the decoder to enrich the semantic information of the shallow features. Most of the current methods concentrate on changing the connection ways between network nodes or changing the structure of convolutional units, ignoring the output characteristics of the convolutional units in the nodes. Tran et al. [40] suggested the Un-Net model based on the traditional U-Net. This approach used the output features of the convolutional units as skip connection and utilized those features from the nodes well. Li and Tso [41] merged the dense module, inception module, and dilated convolution into the original U-Net encoding path, then proposed a bottleneck feature supervision (BSU-Net) model. It achieved Dice per case 96.1% for liver segmentation task and 56.9% for tumor segmentation task. BSU-Net used dilated convolution to expand the perceptual field, but the dilated convolution kernel was discontinuous and failed to cover all image features, which led to loss of image continuity. Wang et al. [42] introduced the idea of recursion into U-Net. The output of the previous state (hidden tensor) and the original image (input image) was cascaded as the input of the next cycle, and the recursive remaining convolutional layer was deployed for feature accumulation to ensure better feature representation in the segmentation task. This kind of lite network has a lesser number of parameters and better real-time performance, but it often brings loss of segmentation accuracy.

### 2.2. Segmentation Based on Edge Information

When we apply the method based on enhanced images to nonenhanced MRI images, the feature maps tend to be blurred near the border of the tumor. This is caused by the unclear tumor boundary in the nonenhanced MRI image. The most direct way to eliminate this kind of blur is to extract more edge information and strengthen the network's attention to the edge. Su et al. [43] designed a continuously expanding boundary-aware network. In this network, the boundary location flow selectively enhanced the characteristics of the boundary. The internal perceptual flow ensured the invariance of the internal features. In order to balance the internal and external information, this method used the transition compensation flow to correct the transition region between the internal and the boundaries. Qin et al. [44] developed a boundary-aware predict-refine architecture BAS-Net. The prediction module was used to predict the saliency maps from the input image. The multiscale residual refinement module refined the saliency maps of the prediction module by learning the residual between the saliency maps and the ground truth. This network can effectively segment fine structures with clear boundaries in natural images, but it is not suitable for medical images with a small number of channels and a single pixel distribution. Chen et al. [45] utilized semantic edge aware loss to implicitly integrate structural information into segmentation prediction. The semantic edge detection network mapped the segmentation mask to the corresponding edge map. Another part of the network, the prediction of segmenting the network output, could be optimized in the embedding space of the semantic edge detection network. These methods are all effective in segmenting fine structures with clear boundaries in natural images, but they are rarely applicable to medical images with a small number of channels, a single pixel distribution, and unclear target boundaries.

In the field of medical image segmentation, there are growing researches focusing on improving the segmentation accuracy of targets by focusing on edges. Seo et al. [46] designed modified U-Net. They added a residual path to the skip connection of U-Net, which contained deconvolution and activation operations. The features in the residual paths were adaptively integrated into the features of the skip connection. In this way, the repetition of low-resolution information of features was avoided; the high-resolution edge information of large targets was extracted more effectively. The edge information of the liver and the morphological information of liver tumor were better processed. This method obtained 89.72% Dice similarity coefficient in the liver tumor segmentation task. The network used MSE as the loss function, and it was computationally simple in the backpropagation process, but it could not adequately capture the structural similarity information of the images. Also, the network has the problem of poor generalization. Oda et al. [20] proposed an edge enhancement segmentation network, which relied on two decoders to restore the original image resolution. One decoder (boundary enhancement) could be used to improve the quality of the segmentation in another decoder (nucleus segmentation). We found that using this additional edge enhancement decoder can effectively predict the edge of the tumor and improve the blur. Nevertheless, it was difficult to distinguish tumor-like tissue in the background. Tang et al. [47] developed a two-stage 2D liver and tumor segmentation framework (E^2^-Net). The first stage was rough segmentation of the liver tumor. The second stage of the edge enhancement network introduced an edge prediction module and used the edge distance map between the liver and the tumor boundary as an additional supervision signal to train the edge enhancement network. The method achieved a Dice coefficient of 82.9% in the liver tumor segmentation task. For enhanced images, the liver is much easier to segment than the tumor, so those two-stage segmentation methods segment the liver first and then the tumor can alleviate the disturbance of background pixels other than the liver. In contrast, for nonenhanced images, the liver cannot be segmented more easily than the tumor. Too much dependence on the segmentation results of the first stage may lead to the performance degradation of the whole model. Segmentation of liver tumor directly can avoid negative optimization between networks.

## 3. Method

In this section, we introduce the overall structure of ECLMS. As shown in Figure 2, localization network and dual-branch segmentation network constitute our model. The localization network generates an accurate map of the lesion location and encodes it into the two-branch segmentation network as guidance information. This information will help the dual-branch segmentation network to improve accuracy. The dual-branch segmentation network is made up of a single-encoder and a dual-decoder structure. The decoder part decodes the border and internal area of the tumor by the two branches, respectively. Since the training objectives of the two branches are consistent, the network can learn more discriminative features, which is helpful to improve the final segmentation performance. Our model involves two types of labels, one of them is called boundary label (marking only the marginal part of the tumor), and the other is called normal label (marking the entire tumor part). Next, we will introduce ECLMS in detail.

### 3.1. Localization Network

The localization network is applied to enhance the capability of locating the tumor of the segmentation network in nonenhanced image data.  Figure 3 shows the network details. We use the classic medical image segmentation network U-Net to generate the rough mask. The information about the location of the tumor is encoded in coarse segmentation mask and utilized to assist the subsequent network in obtaining the exact location of the lesion. Xception [48] follows U-Net to convert location information into location mapping. To strengthen the feature extraction ability and accelerate the convergence of the network, U-Net and Xception are pretrained on MICCAI 2017 LiTS challenge dataset and ImageNet, correspondingly. U-Net is chosen because of its small number of parameters and accurate encoding of image information. Xception is a convolutional network structure entirely based on a separable convolution layer proposed by Google. Separable convolution is a classic approach to reduce the number of convolution parameters, which allows for more efficient use of model parameters. The original image with image-level labels and the coarse segmentation mask obtained from U-Net are concatenated and input to Xception. To extend the resolution of the features, the last max pooling layer of the exit flow was removed by us. After the features pass through the global average pooling (GAP) layer, the softmax activation function maps the outputs of multiple neurons to the [0,1] interval. The class activation mapping (CAM) approach [49] is used to generate class-specific location mappings from the last separable convolutional layer to guide the segmentation network to more accurate predictions.

### 3.2. Dual-Branch Segmentation Network

We innovatively design a dual-branch segmentation network to accurately segment liver tumor, as shown in Figure 4. The encoder part is similar to U-Net, including five double-convolution blocks and four max pooling operations. Each double-convolution block contains two combinations of convolution, and each convolution operation is followed by batch normalization and ReLU. The output feature of the encoder concatenates with the location maps after through the bottleneck multiscale module. Then, enter the two branches of the decoding part, namely, the edge decoding branch and main decoding branch, respectively. Each branch contains four double-convolution blocks and four upsampling. The main decoding branch is used to recover the features of the whole tumor region, and the Mini-UNet at the end is used to extract the edges of the predicted images from the main decoding branch. The edge decoding branch is used to extract the edge features of the tumor and predict the fine boundary. Similar to the dense skip connection of U-Net++, we not only bring in a skip connection between the same scale features of the encoder and the two decoding branches but also concatenate the feature mappings of layers 2, 3, and 4 of the encoder with the same scale features of layers 1, 2, and 3 of the main decoding branch and the edge decoding branch, respectively. And this kind of connection is called dense upward connection. This approach makes the aggregation layer fuse various features carried by the skip connection with the decoder features, enabling the decoder to share the deep features of the encoder. This connection overcomes the limitation that the original skip connection only fuses the same scale features, better recovers the feature information lost in the network during downsampling, and enriches the feature representation of the network. In order to reduce the influence of background interference pixels, we embed channel squeeze and spatial excitation block (sSE block) [22] after each pooling and upsampling operation. It can be added to an existing network without destroying the original main structure of the network. The sSE block mainly includes two parts of channel squeeze and spatial excitation. The squeeze along the channel is achieved through a convolution operation. Spatial excitation is to reactivate the compressed projection tensor to [0,1] with sigmoid function and then multiply the activated weights with the corresponding positions of all channels of the original feature maps. The goal is to recalibrate the feature spatially. This operation increases the weight of important location information in each layer of features. This approach encourages the network to retain more useful information in space and to ignore locations that are not relevant to the tumor region.

### 3.3. Bottleneck Multiscale Module

The bottleneck multiscale module (BMM) consists of three adaptive convolutional blocks (ACB) with different kernel sizes; each of them can acquire the feature representation of a specific scale which is related to the input. Three sizes of convolution kernels are employed in BMM to extract features. These filters are dynamically generated based on the regional context of the input image. This operation can incorporate rich content and high-level semantics and adaptively capture internal variations of the input image, allowing different sized targets to be accurately covered by a single sensory field. This method is more flexible than traditional filters.  Figure 5 shows the internal structure of the BMM.

The input of BMM is the feature maps *x* ∈ *R*^*h*×*w*×*c*^ which is the output of the encoder at the same time. The input feature *x* is processed by 1 × 1 convolution operation to obtain the feature maps *F*(*x*) ∈ *R*^*h*×*w*×*c*′^(*c*′ < *c*), where *h*, *w*, and *c* denote the height, width, and channel number of feature *x*, separately. Adaptive Max Pooling (AMP) can adjust the features to a specified size adaptively. AMP is used to size the feature map *x* to *s* × *s* and then adjust the number of channels by a 1 × 1 convolution to make it equal to the number of channels *c*′*c*′ of *F*(*x*). The generated features are denoted as *K*_*s*_(*x*) ∈ *R*^*s*×*s*×*c*′^. We use *K*_*s*_(*x*) as the convolution kernel to perform a depth-wise convolution operation with the feature *F*(*x*) to obtain a specific scale representation. Different from ordinary convolution operation, depth-wise convolution carries out independent convolution operation on each channel of the input layer. Three scale features after convolution are fused:

(1) $$\begin{array}{c} y_{s}=F\left(x\right)⊗K_{s}\left(x\right), \end{array}$$

(2) $$\begin{array}{c} y^{\prime }=y_{1}⊕y_{3}⊕y_{5}, \end{array}$$

where ⊗ is the convolution operation, ⊕ is the concatenate operation, *s* is the size of the convolution kernel, and *y*_*s*_ ∈ *R*^*h*×*w*×*c*′^ is the output of ACB. We choose *s* = 1, 3, 5 as the three kernel sizes of ACB. We aggregate *y*′, the original feature map *x*, and the location map *M*. The aggregated feature *Y* is input into the edge decoding branch and main decoding branch after 1 × 1 convolution adjustment channel. We will concretely analyze the influence of the number of ACB and convolution kernel size on model performance in the experimental part.

### 3.4. Loss Function

#### 3.4.1. The Location Loss Function

We construct the loss function *L*_loc_ based on Dice loss and rank loss, as well as utilize it to optimize U-Net in the positioning network. First of all, the Dice loss measures the degree of overlap between the prediction and the ground truth. It is suitable for segmentation problems with a small proportion of the foreground. Secondly, pixels which are easy to be classified account for a relatively low proportion of the network optimization process. Hard pixels that are difficult to identify (such as boundary pixels) can provide more information during network learning. For these reasons, we use rank loss to add additional constraints between the boundary pixels of the tumor region and the background. This loss can help the network focus on learning more discriminative information in hard pixels. *L*_loc_ is defined as

(3) $$\begin{array}{c} L_{\text{loc}}=1-\frac{2\sum_{i}\alpha_{i}\beta_{i}+\text{smooth}}{\sum_{i}\alpha_{i}+\sum_{i}\beta_{i}+\text{smooth}}+\lambda_{1}\frac{\sum_{i=1}^{K}\sum_{j=1}^{K}\max\left\{0,B_{i}^{n}-T_{j}^{n}+\mu \right\}}{K^{2}}, \end{array}$$

where the first item is Dice loss. *α*_*i*_ denotes the probability that pixel *i* is classified as tumor area. *β*_*i*_ means the ground truth of the corresponding area. The parameter smooth is used to avoid the denominator being 0. Here, we set smooth = 1*e* − 5. *λ*_1_ is a weighting factor that balances these two losses. *n* denotes the *n*^th^ input image. *K* denotes the *K* pixels with the largest error in the tumor area or the background area. *B*_*i*_^*n*^ and *T*_*j*_^*n*^ denote the predicted values of the *i*^th^ hard pixel of the background and the *j*^th^ hard pixel of the tumor. After each batch of forward propagation, the pixels of the lesion and the background area are sorted according to the error.

#### 3.4.2. The Segmentation Loss Function

The goal of *L*_seg_ is to reduce the difference between the ground truth with prediction masks and the boundary predictions generated by the edge decoding branch and the main decoding branch, respectively. It consists of multiple independent losses, which are the area loss *L*_area_, the edge loss *L*_edge_, the edge detection loss *L*_ed_, and the constraint loss *L*_con_. These losses are defined in detail as follows:

(4) $$\begin{array}{c} L_{\mathrm{seg}}=L_{\text{area}}+L_{\text{edge}}+L_{\text{ed}}+\lambda_{2}L_{\text{con}},\\ L_{\text{area}}=-\underset{i}{\sum }x_{i}\log\left(\alpha_{i}\right)+\left(1-\frac{2\sum_{i}\alpha_{i}\beta_{i}+\text{smooth}}{\sum_{i}\alpha_{i}+\sum_{i}\beta_{i}+\text{smooth}}\right),\\ L_{\text{edge}}=-\underset{i}{\sum }y_{i}\log\left(p_{i}\right),\\ L_{\text{ed}}=-\underset{i}{\sum }y_{i}\log\left(q_{i}\right),\\ L_{\text{con}}=-\underset{i}{\sum }p_{i}\log\left(\frac{q_{i}}{p_{i}}\right)-\underset{i}{\sum }q_{i}\log\left(\frac{p_{i}}{q_{i}}\right), \end{array}$$

where *L*_area_ measures the difference between the output of the main decoding branch and the normal label. The crossentropy loss function penalizes pixel classification errors. The Dice loss function measures the degree of overlap between the predicted tumor area and the normal label, which can alleviate the imbalance between the target and the background. *L*_edge_ supervises the edge decoding branch output, where *p*_*i*_ represents the probability that the pixel *i* is the tumor boundary, and *y*_*i*_ ∈ {0, 1} is the corresponding boundary label. The purpose of *L*_ed_ is to minimize the difference between the output of the boundary detector (Mini-UNet) and the boundary label, where the result is predicted by Mini-UNet. The constraint loss *L*_con_ is for establishing dependencies between the main decoding branch and the edge decoding branch to prevent them from deviating from each other. For the hyperparameters in the loss function, we separately set *λ*_1_ = 0.05, *λ*_2_ = 0.5, *K* = 30, and *μ* = 0.3.

## 4. Experiment

### 4.1. Dataset

Our nonenhanced MRI dataset is composed of 215 different subjects (130 subjects with hepatic hemangioma and 85 subjects with hepatocellular carcinoma). For each of our data, an informed permission for data use is obtained and signed by the patient. Three lesion images are chosen for each case to obtain 645 liver tumor images. Each subject has undergone a standard clinical liver MRI examination and collected liver axial MRI images by a GE Signa HDx 3.0 T MRI System. T1WI modality is mainly applied to observe the anatomical structure of organs and tissues. In T2WI modality, the accumulation of water molecules results in a higher signal than the surrounding normal tissue. Therefore, T2WI is better for finding lesions. This paper uses T2WI (256 × 256 px) as training and test data and randomly initializes the weights of the dual-branch segmentation network. In order to ensure the consistency of boundary label and normal label, the boundary label is first marked to obtain the boundary label, and then, the boundary label is filled to obtain the normal label. We select 80% of all data as the training set and 20% as the test set and used 5-fold cross-validation to evaluate the model. Then, we augment the data of the training set by rotating each image horizontally by 90°, 180°, and 270° and scaling outward by 50% with the location of the tumor in the center. The final dataset after data augmentation contains a total of 2709 images (2580 in the training set and 129 in the test set).

### 4.2. Evaluation Metrics

We utilize three standard metrics, Dice similarity coefficient (DSC), pixel accuracy, and precision to evaluate our model, where TP, FP, TN, and FN are divided into true positive, false positive, true negative, and false negative. The Dice similarity coefficient is the most commonly measured evaluation metrics in segmentation networks. It is adopted to measure the spatial overlap accuracy between the network segmentation result and the golden standard mask in the field of image segmentation. DSC is defined as follows:

(5) $$\begin{array}{c} \text{DSC}=\frac{2\text{TP}}{\text{FP}+2\text{TP}+\text{FN}}. \end{array}$$

Pixel accuracy is a common and intuitive evaluation index, which represents the proportion of pixels that are correctly predicted to the total pixels. It is usually expressed as

(6) $$\begin{array}{c} \text{Accuracy}=\frac{\text{TP}+\text{TN}}{\text{TP}+\text{TN}+\text{FP}+\text{FN}}. \end{array}$$

Precision represents the proportion of pixels predicted to be tumor to the actual tumor pixels. It focuses on judging whether the predicted mask accurately covers the tumor area. The precision is defined as

(7) $$\begin{array}{c} \text{Precision}=\frac{\text{TP}}{\text{TP}+\text{FP}}. \end{array}$$

### 4.3. Implementation Details

The deep learning framework used in our experiment is PyTorch (version 1.4.0). The CUDA version is 10.1. We implement our network on a 1.90 GHz Intel(R) Xeon(R) E5-2620 CPU and NVIDIA TITAN XP GPU computer. Stochastic gradient descent (SGD) optimizer is applied to update the network parameters of ECLMS. We set the momentum to 0.9, weight decay to 0.0005, initial learning rate to 0.001, batch size to 8, and epoch to 500.

### 4.4. Ablation Study

To further evaluate our model, we conduct ablation experiments under different settings. Each time we introduce a modification to measure our contribution to the overall improvement of the model, we analyze the impact of the network that generates the location map, the embedding location of the sSE block, and some important hyperparameters on the model results. We combine all indicators to determine the most suitable configuration. The best results in each experiment are shown in italic.

#### 4.4.1. Ablation for sSE Block

We analyze the impact of the embedding position of sSE block on the performance of the model.  Table 1 reports the results of adding sSE blocks in different locations. For the convenience of presentation, we replace main decoding branch and edge decoding branch with Mdb and Edb. After embedding sSE blocks in both the encoding part and the decoding part, the model reaches the highest level in Dice and accuracy. The difference between precision and the highest score is only 0.14%. On the whole, embedding sSE block in the main decoding branch and edge decoding branch has the greatest improvement in model performance. We believe that the constraint loss between the two branches converges their prediction results. If sSE block is embedded in one branch alone, it will aggravate the prediction difference between the two branches, and the prediction accuracy of the branch with accurate prediction will be pulled down by the other one with inaccurate prediction, resulting in a worse overall performance.

#### 4.4.2. Ablation for BMM

In this experiment, we test the effects of different adaptive convolutional block (ACB) numbers and different sizes of convolution kernel in the BMM on the performance of the module. We try three cases where the number of ACB is 2, 3, and 4. Each ACB number corresponds to the combination of different core sizes. We choose four common kernel sizes of 1, 3, 5, and 7 to achieve different combinations. In Table 2, BMM shows the best performance when the ACB number is 3 and the kernel size is 1, 3, and 5. Dice, precision, and accuracy are increased by 3.69%, 4.25%, and 4.48%, respectively. When the convolution kernel is increased to 7 × 7, the network performance incurred decay. This is because a large size of convolution kernel like 7 × 7 brings a larger perceptual field while losing more image details, and the loss of this detailed information for tumor of smaller size leads to a degradation of the model performance. Also, large-size convolution adds more parameters and computational complexity.

#### 4.4.3. Ablation for Hyperparameter of Loss Function

We perform ablation experiments for the four hyperparameters (*λ*_1_, *λ*_2_, *K*, and *μ*) in the loss function to determine their optimal values. We evaluate the performance of different values of hyperparameters on three evaluation metrics and select the highest evaluation metric that can be obtained as the optimal set of hyperparameters. As shown in Figure 6, the three evaluation metrics Dice, precision, and accuracy reach the highest level when *λ*_1_ = 0.05, *λ*_2_ = 0.5, *K* = 30, and *μ* = 0.3.

#### 4.4.4. Ablation for Localization Network

We choose VGG16 [50] and the three revolutionary architectures ResNet50 [51], Inception v3 [52], and Xception in the neural network as candidate networks for generating location mapping. VGG16 is a common convolutional neural network. It is composed of several convolutional layers and pooling layers in a stacked manner. Each block of ResNet is composed of a series of layers and a shortcut connection. This shortcut causes the gradient to backpropagate to the previous layer, ensuring that the network of layer *l* + 1 contains more image information than layer *l*. Then, perform the add operation on the element level. In Inception v3, input data is mapped to multiple smaller input spaces using 1 × 1 convolution. For each of these input spaces, a different type of filter is used to perform transformations on smaller modules of these data. Xception maps the spatial correlation separately for each output channel and then uses 1 × 1 depth-wise convolution to extract crosschannel correlation. All four models are initialized with weights pretrained on ImageNet.  Table 3 is the comparison result of using these four kinds of networks. The comparison results show that the network using Xception shows the best performance. As the result, we use Xception in ECLMS to generate location mapping.

#### 4.4.5. Ablation for the Contribution of Each Component

We test the performance of the model while gradually reducing the components. Different components have different degrees of performance contribution to the model. The quantitative analysis results are shown in Table 4. We abbreviate the localization network as L-Net in the figure and table. The comparison results show that sSE block, BMM, and localization network all have a certain degree of gain in segmentation network performance.

In Figure 7, we visualize the segmentation results and corresponding location mappings with and without localization network on the three cases of data. It can be seen that location maps focus the attention of the network around the tumor. Compared with only using the dual-branch segmentation network, the model can better reduce the interference of background pixels after adding the positioning network and achieve better performance. This proves that the use of location mapping to assist the segmentation of noncontrast images is crucial.

### 4.5. Comparison to State of the Art

We compare the performance of the proposed ECLMS model with existing segmentation methods to show the advancement of our method. The comparison methods are (1) U-Net, (2) U-Net++, (3) BESNet, and (4) RgGAN, where U-Net is a classic method in medical image segmentation; U-Net++ is an improved method based on U-Net; BESNet is a dual decoder network based on boundary enhancement; and RgGAN is the latest liver tumor segmentation method based on GAN without contrast agent. To ensure the fairness of the experiments, the comparison experiments between the method in this paper and the remaining four methods are completed in the same hardware environment and dataset. The comparative results are shown in Table 5. Our method obtains the best results on the three evaluation metrics. ECLMS achieves 90.23 ± 2.01% in Dice, 92.25 ± 1.97% in precision, and 92.39 ± 1.88% in accuracy.

In Figure 8, we visualize the other methods and our method segmentation results of five cases of data. The results show that the first three methods are greatly affected by background pixels and cannot accurately locate tumors that are difficult to identify with the naked eye. Our ECLMS, however, enables the network to better identify the tumor region due to the incorporation of location mapping, which effectively reduces the interference of background spoof pixels and allows more accurate localization of the tumor. Since RgGAN introduces the radiomic characteristics of the tumor as prior knowledge, the segmentation effect has been significantly improved, but the prediction of the tumor boundary is not accurate enough. Our method uses an edge decoding branch to predict tumor edge pixels, allowing fuller capture of detailed information of tumor edges. Also, sSE block spatially increases the weight of important features to make the network provide more attention to the tumor region. Our method effectively reduces the interference of background deception pixels and obtains a smoother tumor edge. At the same time, the segmentation accuracy of small tumor is improved.

### 4.6. Model Complexity Analysis

We compare ECLMS with four existing methods in the area of the number of model parameters. The most common measure of model complexity is parameter count (Params).  Table 6 shows our statistical results. From the results, the number of parameters for our method is much smaller than that of RgGAN which is the latest nonenhanced image segmentation method with better generalization. The number of parameters of our method is larger than that of the first three methods, because of the targeted optimization made by our method for nonenhanced images of the liver. The models with lower complexity (such as the first three models) can barely reflect the complex spatial and detailed information of nonenhanced MRI and have lower segmentation accuracy.

## 5. Conclusion and Future Work

This paper proposes a novel liver tumor segmentation model based on edge constraint and location mapping for nonenhanced MRI. The localization network is used to generate a location mapping that is capable of assisting the dual-branch segmentation network to locate the tumor. The dual-branch segmentation network can decode the internal and boundary features of the tumor at the same time, and the rich edge features can effectively enhance the network's ability to recognize fuzzy boundaries. We embed the sSE module in the network, which can automatically obtain the importance of each feature channel by self-learning. We also enrich the shallow features of the network by introducing dense skip connection. The bottleneck multiscale module after the encoder acquires a multiscale feature representation of the image by using different sizes of convolutional kernels. The location mapping generated by the localization network is also fused to improve the perceptual dimensionality of the network. Our ECLMS achieves 90.23%, 92.25%, and 92.39% on Dice, precision, and accuracy, respectively. These results prove that it is an effective computer-aided diagnosis tool. Our ECLMS has significant advantages for medical images with blurred edges and can help radiologists segment liver tumor in the absence of contrast agent.

Although this paper emphasizes the potential and applicability of the ECLMS model in nonenhanced image segmentation, there are still some questions that deserve our continued research. (1) When the location mapping is fused to the segmented network, we only carry out simple concatenate operation between the output feature and the location mapping, which may lead to insufficient utilization of the location information in such a direct stitching way. In the future, we will try new integration methods to address this shortcoming. (2) Since the 2D method only encodes in two directions and cannot obtain the interlayer context information of the sequence images, our future work considers extending ECLMS to 3D. The 3D network utilizes more abundant information in the *z*-axis direction and can fully capture the context information between layers and restore the target features more continuously in the three-dimensional space. However, due to the matching problem between the amount of data and the amount of model parameters, the 3D network may need more data to train, otherwise it will lead to overfitting.

## Figures and Tables

**Figure 1:** (a) Shows the nonenhanced images and enhanced images before and after contrast injection in two patients. The nonenhanced images have low contrast between the tumor region and tissues; the tumor edges are also blurred. (b) Demonstrates that there is not only diversity in morphology and size of liver tumor in the nonenhanced images but also many tumor-like tissues that are cheating.

**Figure 2:** Our ECLMS model is composed of localization network and dual-branch segmentation network. The tumor location maps generated by the localization network, which is used as the guide information to be fused into the segmentation network. The main decoding branch and edge decoding branch in dual-branch segmentation network can be mutually restrained and jointly optimized in the direction of ground truth.

**Figure 3:** The structure of location network.

**Figure 4:** The structure of dual-branch segmentation network.

**Figure 5:** The bottleneck multiscale module uses adaptive convolutional blocks with convolutional kernel sizes of 1, 3, and 5 to extract multiscale features and concatenate the extracted features with location mappings.

**Figure 6:** Comparison results for different values of the hyperparameters in the loss function.

**Figure 7:** Comparison of segmentation results with and without localization network.

**Figure 8:** Comparison of segmentation masks is generated by different methods. (a–d) Are the segmentation results of the other four methods; (e) is the segmentation results of our model; (g) shows the nonenhanced images and tumor details. We mark the ground truth with a red box, and the segmentation results with inaccurate positioning or poor effect are marked with a blue box.

**Table 1:** Comparison results of sSE block embedding in different positions.

Location of sSE blocks	Dice (%)	Precision (%)	Accuracy (%)
Without sSE blocks	85.03 ± 1.37	89.13 ± 1.66	87.65 ± 0.98
Only encoder	86.31 ± 1.45	87.55 ± 1.22	88.28 ± 0.69
Encoder + Edb	87.64 ± 2.07	89.79 ± 1.35	88.72 ± 2.09
Encoder + Mdb	88.18 ± 1.98	91.52 ± 1.48	91.46 ± 1.62
Encoder + Mdb + Edb	88.72 ± 1.27	91.38 ± 1.03	92.01 ± 0.76
Encoder + Mdb + Edb + Mini‒UNet	86.01 ± 2.63	90.23 ± 2.24	89.94 ± 1.57

**Table 2:** Comparison results of using different numbers of ACB and size of convolution kernel.

ACB number	Kernel size	Dice (%)	Precision (%)	Accuracy (%)
0	—	85.03 ± 1.37	87.13 ± 1.66	87.53 ± 0.98
2	1, 3	85.33 ± 1.35	88.72 ± 2.57	89.46 ± 2.21
2	3, 5	87.67 ± 1.28	88.42 ± 1.49	91.32 ± 1.77
3	1, 3, 5	88.72 ± 1.27	91.38 ± 1.03	92.01 ± 0.76
3	3, 5, 7	87.92 ± 1.52	89.65 ± 2.13	90.11 ± 0.89
4	1, 3, 5, 7	87.26 ± 1.21	88.39 ± 1.33	90.31 ± 1.71

**Table 3:** Comparison results of four candidate networks for generating location mapping.

Network	Dice (%)	Precision (%)	Accuracy (%)
VGG16	86.52 ± 1.74	88.46 ± 2.10	90.35 ± 2.44
ResNet50	89.75 ± 1.83	90.18 ± 1.36	91.24 ± 2.31
Inception v3	88.31 ± 2.45	92.03 ± 2.62	91.48 ± 1.79
Xception	90.23 ± 2.01	92.25 ± 1.97	92.39 ± 1.88

**Table 4:** Performance comparison results of gradually reducing components.

Models	Dice (%)	Precision (%)	Accuracy (%)
ECLMS	90.23 ± 2.01	92.25 ± 1.97	92.39 ± 1.88
ECLMS − L‒Net	88.72 ± 1.27	91.38 ± 1.03	92.01 ± 0.76
ECLMS − BLNet − BMM	87.30 ± 2.07	91.02 ± 1.64	90.86 ± 1.24
ECLMS − BLNet − BMM − sSE	84.21 ± 2.26	89.17 ± 1.79	87.39 ± 2.86

**Table 5:** Comparison results with existing segmentation methods.

Methods	Year	Dice (%)	Precision (%)	Accuracy (%)
U-Net	2015	77.31 ± 1.19	82.88 ± 0.75	83.66 ± 1.24
U-Net++	2019	84.51 ± 2.37	85.36 ± 3.62	84.03 ± 2.02
BESNet	2018	83.69 ± 1.85	86.44 ± 2.47	87.23 ± 3.26
RgGAN	2019	88.09 ± 2.67	89.16 ± 1.34	91.92 ± 2.15
Our method	2021	90.23 ± 2.01	92.25 ± 1.97	92.39 ± 1.88

**Table 6:** Results of model complexity comparison with existing segmentation methods.

Methods	Params (M)	Dice (%)
U-Net	7.8	77.31 ± 1.19
U-Net++	9.0	84.51 ± 2.37
BESNet	15.4	83.69 ± 1.85
RgGAN	95.8	88.09 ± 2.67
Our method	51.9	90.23 ± 2.01

## Data Availability

The datasets of images used to support the findings of this study are available from the corresponding author upon request.
